The article "Study on Automatic Multi-Classification of Spine Based on Deep Learning and Postoperative Infection Screening" was retracted in 2023. Reasons: signs of a paper mill; suspected computer-generated content; unreliable results or conclusions; lack of ethics approval or compliance.

# Study on Automatic Multi-Classification of Spine Based on Deep Learning and Postoperative Infection Screening

**DOI:** 10.1155/2022/2779686

**Published:** 2022-03-22

**Authors:** Hua Wang, Yanxiao Liu, Yancheng Li

**Affiliations:** Department of Orthopedics, Quzhou People's Hospital, Quzhou, Zhejiang 324000, China

## Abstract

The preoperative qualitative and hierarchical diagnosis of intervertebral foramen stenosis is very important for clinicians to explore the effect of multimodal analgesia nursing on pain control after spinal fusion and to formulate treatment strategies and patients' health recovery. However, there are still many problems in this aspect, and there is a lack of relevant research and effective methods to assist clinicians in diagnosis. Therefore, to improve the accuracy of computer-aided diagnosis of intervertebral foramen stenosis and the work efficiency of doctors, a deep learning automatic grading algorithm of intervertebral foramen stenosis image is proposed in this study. The image of intervertebral foramen was extracted from the MRI image of sagittal spine, and the image was preprocessed. 86 patients with spinal fusion treated in our hospital, specifically from May 2018 to May 2020, were randomly divided into the control group (routine analgesic nursing) and the multimodal group (multimodal analgesic nursing), with 43 cases in each group. The pain control effect and satisfaction of the two groups were observed. The results after multimodal analgesia nursing show that the VASs of the multimodal group at different time points were significantly lower than those of the control group (*P* < 0.05); the satisfaction score of pain control in the multimodal group was significantly higher than that in the control group (*P* < 0.05). Multimodal analgesia nursing for patients undergoing spinal fusion can effectively reduce the degree of postoperative pain and improve the effect of pain control and satisfaction with pain control, which is worthy of promotion.

## 1. Introduction

Spinal fusion is an effective way to treat lumbar diseases in clinic, but the spine is the pillar of the body. Spinal surgery has great trauma, and patients usually need to bear unbearable pain after operation. If the analgesia is insufficient, it is very easy to increase the occurrence of postoperative complications and delay the process of postoperative rehabilitation [1]. Therefore, it is very important to strengthen the pain management after spinal fusion. Opioids are common analgesics. Although they have certain analgesic effects, the use of opioids alone in large doses is easy to produce drug tolerance, accompanied by many adverse reactions, resulting in low pain control effect and control satisfaction [2]. The application and development of multimodal analgesia nursing provide an effective guarantee for clinical analgesia nursing. In recent years, it has been gradually applied to various surgical analgesia and achieved satisfactory results [3].

The article "Study on Automatic Multi-Classification of Spine Based on Deep Learning and Postoperative Infection Screening" was retracted in 2023. Reasons: signs of a paper mill; suspected computer-generated content; unreliable results or conclusions; lack of ethics approval or compliance.

Intervertebral foraminal stenosis (IFS) is a degenerative disease caused by intervertebral foraminal stenosis compressing the peripheral nervous system of spinal nerve roots [4]. As the transmission center of sensory input, the spinal nerve root will cause pain, muscle weakness, and even physical disability after being compressed, and IFS will lead to severe scoliosis and spondylolisthesis with the natural aging process of people. About 80% of the elderly are suffering from low back pain caused by IFS [5]. Clinical data show that the treatment plan varies with IFS grade. For example, for grade 1 stenosis, general physical therapy and exercise will be the first choice for treatment, while for more severe grade, patients may need surgical treatment or decompression treatment [6]. Therefore, effective and accurate grading is a crucial step in the diagnosis and treatment of intervertebral foramen stenosis. However, the existing clinical classification of intervertebral foramen stenosis mainly has three problems: (1) the visual inspection and manual scoring of IFS images by doctors are time-consuming, labor-consuming, and inefficient; (2) due to the diversity of IFS, clinicians often pay more attention to intervertebral disc herniation, spinal canal stenosis, and lateral recess stenosis, but tend to ignore the stenosis of intervertebral foramen, which is highly subjective; and (3) the special anatomical structure of intervertebral foramen and complex stenosis causing factors are easy to make it difficult to judge comprehensively and accurately, and the rate of misdiagnosis and missed diagnosis is high. Therefore, to improve the diagnostic efficiency of IFS, the subjective influence of doctors is reduced and the rate of misdiagnosis and missed diagnosis is reduced, and the design of automatic clinical auxiliary diagnostic system has important application value [7].

At present, important progress has been made in the research of computer-aided diagnosis of IFS, which can be divided into two types according to different regions of interest. The first type is the research on automatic location and segmentation based on the structure around the intervertebral foramen. Reference [8] used a two-level model to capture pixel-level and object-level features in MRI images to realize the local anomaly detection of intervertebral discs; [9] used a common spine geometry design and analysis algorithm based on CT and MR images to initialize the marking of vertebrae to realize vertebral positioning; [10] used regression segmentation method to segment M3 spine map. The second type is the automatic segmentation or grading research directly based on the intervertebral foramen. Reference [11] realized the segmentation by detecting the center line of the vertebral body and the main boundary points of the intervertebral foramen; [12] used the AdaBoost detection algorithm and iterative normalization segmentation algorithm to detect MRI vertebral body images and locate and segment them at the same time; [13] realized the modeling and segmentation of spine and intervertebral foramen based on two scales by representing the global spine shape in a continuous local vertebral coordinate system and modeling the individual vertebrae as a triangular surface network; [14] used the super-pixel segmentation method to achieve an accuracy of 98.52% in the image location and benign and malignant classification of intervertebral foramen stenosis.

The article "Study on Automatic Multi-Classification of Spine Based on Deep Learning and Postoperative Infection Screening" was retracted in 2023. Reasons: signs of a paper mill; suspected computer-generated content; unreliable results or conclusions; lack of ethics approval or compliance.

The above studies have made varying degrees of progress, but there are still some problems. This kind of auxiliary diagnostic research based on partial morphological and anatomical structure localization, segmentation, or simple secondary classification ignores the global information and affects the diagnostic accuracy. Clinically, the diagnosis of intervertebral foramen stenosis based on conventional supine MRI images is determined by many factors such as intervertebral foramen morphology, periradicular fat, or morphological changes in nerve roots. For example, although grade 2 stenosis has no morphological changes in four directions (vertical and transverse) around nerve roots, intervertebral disc space stenosis, and ligament macular thickening, small joint disease and intervertebral disc herniation also lead to nerve root compression, which is easy to be misdiagnosed [15]. Therefore, the study of an efficient algorithm to extract the global “lesion features” of the image and realize automatic hierarchical diagnosis has become an important problem to be solved in auxiliary IFS diagnosis. In terms of image processing algorithms, the deep learning model can well extract the deep features of the image and can reduce the feature redundancy and improve the feature correlation by changing the network topology of the model, such as appropriately increasing the depth and width of the network. Since [16] applied a convolutional neural network to medical image analysis in 1995, the deep learning model has rapidly become an important method for studying and analyzing medical images [17], and it has made important progress in assisting the clinical diagnosis of brain, breast, lung, and other organs, but the research on assisting the diagnosis of spinal diseases is basically blank.

The article "Study on Automatic Multi-Classification of Spine Based on Deep Learning and Postoperative Infection Screening" was retracted in 2023. Reasons: signs of a paper mill; suspected computer-generated content; unreliable results or conclusions; lack of ethics approval or compliance.

In this study, a deep learning automatic grading algorithm of intervertebral foramen stenosis image is proposed to improve the accuracy of computer-aided diagnosis of intervertebral foramen stenosis and the work efficiency of doctors. The image of intervertebral foramen was extracted from the MRI image of sagittal spine and was preprocessed. The main contributions of this study are as follows:

1. A supervised deep convolutional neural network, which is based on automatic classification of intervertebral foraminal stenosis (IFS net), is designed and developed to extract image texture features, color features, shape features, and spatial relationship features.
2. Various characteristics, which are extracted through the proposed model, serve as the “symptom” characteristics of different levels of disease to establish a special “pathological” relationship with IFS.
3. Additionally, advanced transfer learning and fine-tuning methods are adopted to resolve the issues of large amount of training data and the number of IFS image data.

The rest of the study is organized as given in the following paragraph.

In Section 2, a thorough evaluation of the existing state-of-the-art methods, which is based on their performance in resolving the aforementioned, is presented, which is followed by the proposed model development and implementation plan. The experimental results are presented in Section 4. Finally, concluding remarks are provided in the last section of the manuscript just before references.

## 2. Related Work

With the rapid development of science and technology, artificial intelligence has become a keyword in recent years and has been widely used in all walks of life. The field of medical and health is one of its important application scenarios. With the national attention to medical undertakings, the amount of clinical medical data increases exponentially, and the traditional medical diagnostic methods cannot meet the needs of modern society. This study aimed to point out the development direction of intelligent medicine in the future using the example of the integration of machine learning and medical field.

The world is turned upside down in computer mobile phone. The incidence rate of some diseases is increased. More and more people either sit in front of the computer for a long time or “bow their heads” on mobile phones, resulting in spinal diseases, vision loss, and other health problems. Among them, spinal-related diseases are the first of all diseases endangering human health. It will lead to various diseases such as heart disease and cerebral infarction and even cause paralysis and death of lower limbs. Early diagnosis and treatment are the key to improve the cure rate of spinal diseases, which needs a good medical security system and advanced medical technical support. As we all know, the development of the medical field is based on science and technology. In recent years, with the continuous promotion of artificial intelligence technology and the continuous growth of medical service demand, the society urgently needs medical intelligence. “Artificial intelligence + medical” will become an important driving force to solve the shortage of medical resources and improve the production in the medical field. The intelligent diagnosis of this study is to use artificial intelligence technology in auxiliary diagnosis and treatment, use the medical data set to let the computer “learn” the medical knowledge of professional doctors, simulate doctors' thinking and diagnostic reasoning, and give reliable diagnostic results.

The article "Study on Automatic Multi-Classification of Spine Based on Deep Learning and Postoperative Infection Screening" was retracted in 2023. Reasons: signs of a paper mill; suspected computer-generated content; unreliable results or conclusions; lack of ethics approval or compliance.

Intelligent diagnosis and treatment are the most important and core application scenario of artificial intelligence in the medical field, which has broad development prospects. In the application of “artificial intelligence + medical treatment,” the Watson system of IBM is a relatively mature case in the world IBM. Watson integrates machine learning with traditional medical diagnostic model to provide processing logic ability of intelligent auxiliary diagnosis and treatment. In December 2017, Zhejiang Hospital of Traditional Chinese Medicine, together with Sichuan Yihui and Hangzhou Cognitive Network Technology Co., Ltd., established the Watson joint consultation center, which means that the commercial trial application of the Watson intelligent diagnosis and treatment in China's medical field has been officially implemented.

## 3. Proposed Mechanism or Model

### 3.1. Algorithm Structure

IFS net designed in this study is an end-to-end pattern recognition model, which can realize the high-precision automatic classification of IFS, and has the characteristics of simple and efficient network structure. The end-to-end method enables the model to automatically feedback the loss value to each layer while extracting the potential features of the image and adjusts the model parameters for many iterations to obtain the optimal solution. IFS net model structure includes 8 layers of network structure, including 3 convolution layers, 3 pooling layers, 1 full-connection layer, and 1 output layer, of which the full-connection layer and the output layer are the advantageous modules of the model, so as to maximize the use of the feature information extracted by the model, so as to achieve more effective classification. The IFS net model framework is shown in Figure 1. The main structure and functions include the following.

(1) Input Layer: this layer introduces the whole intervertebral foramen image into the IFS net structure and generates the input of the first convolution layer.
(2) Convolution Layer: this layer is responsible for feature learning. This layer extracts features by convolution calculation of the output of neurons connected to the local area of the input layer or the upper layer. Each neuron is connected to the area of the previous layer as a sparse connection. The weight set of input convolution is convolution kernel, also known as filter. A learnable convolution kernel is convoluted with several feature maps in the previous layer. After accumulating all elements and adding a bias, it is transmitted to a nonlinear activation function. The structure of this study uses ReLU function as the nonlinear activation function. In addition, to reduce the computational complexity, the connection weights between some neurons in the same layer are shared, that is, the same. The size of each layer of filter decreases in turn, which is 7 × 7, 5 × 5, and 3 × 3. The step size is set to 2; it is initialized by the Gaussian distribution, and the standard deviation is 0.01. The three convolution layers contain 32, 64, and 128 feature maps, respectively. The convolution calculation formula is shown as follows:
  (1) $$\begin{array}{c} x_{K_{j}}^{l}=f\left(\left(\underset{ieM^{M-1}}{\sum }x_{i}^{i-1}*K_{ij}^{l}\right)+b_{j}^{l}\right), \end{array}$$
  where *l* represents the number of layers; *K*_*ij*_^*l*^ represents the convolution kernel connecting the feature map of layer *L* and the feature map of layer L−1; *M*^*L*−1^ represents the input feature maps selected by the L−1 layer; *∗* represents convolution operation; *b*_*j*_^*l*^ represents the offset of map in *L* layer; and *f*(.) represents the nonlinear activation function.
(3) Pooling layer: the purpose of the pooling layer is to reduce the dimension of feature maps by reducing similar feature points. In addition, it can also reduce noise and expand the acceptance domain [18]. The output of the pooling layer reduces the number of parameters while keeping the scalar unchanged. The three pooling layers of the model in this study adopt the strategies of max pooling and mean pooling to realize feature dimensionality reduction, with a step size of 2. The pooling layer has the same number of feature maps as its front-end volume layer, which are 32, 64, and 128, respectively.
(4) Full-connection layer: there are 512 neural units in this layer, and each neural unit is fully connected with the upper layer to finally obtain 512-dimensional feature vector.
(5) Output layer: the output layer is composed of European radial basis function (e-rnf) units. The calculation formula is as follows:

(2) $$\begin{array}{c} y_{j}=\sum_{j}|{\left(x_{i}-w_{ij}\right)}^{2}, \end{array}$$

where *x*_*i*_ and *w*_*ij*_ are the input and weight of the last convolution layer, respectively.

The article "Study on Automatic Multi-Classification of Spine Based on Deep Learning and Postoperative Infection Screening" was retracted in 2023. Reasons: signs of a paper mill; suspected computer-generated content; unreliable results or conclusions; lack of ethics approval or compliance.

In addition, the learning rate of the model is 0.000 1, the maximum number of iterations is 25000, the momentum is set to 0.9, and the stochastic gradient descent (SGD) is selected as the optimization function.

### 3.2. Algorithm Training Strategy

#### 3.2.1. Parameter Initialization

In terms of parameter weight initialization of IFS net model, this study adopts the parameter initialization strategy of the combination of self-training and transfer learning. The self-training method is to train the model from scratch by randomly initializing the network parameters; the transfer learning method uses the pre-trained parameter weight to initialize the network, so that the model learns the most basic features (such as color and edge features) in advance, which can help to classify the target data set and improve the classification performance of the algorithm. Random initialization of network parameters is the most commonly used deep learning training method, but considering that one limitation of deep learning in medical image processing is that the size of data set cannot be maximized. Therefore, to improve the classification accuracy and solve the overfitting problem of deep learning algorithm on the small sample data sets, this study uses the method of reference [19] to apply transfer learning to this algorithm.

The main principle of transfer learning is that there is a source domain *D*_*s*_={*X*_*s*_, *P*_*s*_(*X*_*s*_)} with task *T*_*s*_={*Y*_*s*_, *f*_*s*_(.)} and a target domain *D*_*t*_={*X*_*t*_, *P*_*t*_(*X*_*t*_)} with task *T*_*t*_={*Y*_*t*_, *f*_*t*_(.)}. The conditions between the domain and the task are *D*_*s*_ ≠ *T*_*i*_ and *T*_*s*_=*T*_*t*_. In transfer learning, the “knowledge” obtained by *T*_*s*_ and *D*_*s*_ is used to help the learning of prediction function *D*_*t*_ in *f*_*t*_(.). One domain consists of feature space and edge probability distribution. *T*_*s*_ and *D*_*s*_ are the tasks and domains of model training other data sets, and *D*_*t*_ and *T*_*t*_ are the training tasks and domains of this study.

In this study, the model is pre-trained on the ImageNet data set, and then, the obtained network parameters are migrated to the target data set for training, so as to obtain stable network parameters. The data set contains more than 120 natural images and more than 1000 different categories.

The article "Study on Automatic Multi-Classification of Spine Based on Deep Learning and Postoperative Infection Screening" was retracted in 2023. Reasons: signs of a paper mill; suspected computer-generated content; unreliable results or conclusions; lack of ethics approval or compliance.

#### 3.2.2. Softmax Classifier

The model uses softmax classifier to quantify the probability of the “distributed features” extracted by the model. For the training set {(*x*^(1)^, *y*^(1)^), (*x*^(2)^, *y*^(2)^),…, (*x*^(*m*)^, *y*^(*m*)^)}, the corresponding label is *y*^(*i*)^ ∈ {1,2,…, *k*}, which is set here. For each input, there is a corresponding probability of each class.

The model uses softmax classifier to quantify the probability of the “distributed features” extracted by the model. Softmax is the generalization of logistic regression two classifiers to multi-classification. For the training set, the corresponding label is set here. For each input, there is a corresponding probability of each class, that is, the softmax function:

(3) $$\begin{array}{c} P\left(j\right)=\frac{\exp\left(\theta_{i}^{T}x\right)}{\sum_{i=1}^{k}\exp\left(\theta_{i}^{T}x\right)}, \end{array}$$

where *θ*_*i*_^T^*x* is the input from the most sufficient layer to the output layer and is the softmax parameter. Training optimization is essentially a process of approaching the best *θ*^*T*^. Then, the loss function of softmax is as follows:

(4) $$\begin{array}{c} J\left(\theta \right)=-\frac{1}{m}\left[\sum_{i=1}^{m}\sum_{j=1}^{k}1\left\{y^{\left(i\right)}=j\right\}.\;\log\left(P\left(j\right)\right)\right], \end{array}$$

where 1{*y*^(*i*)^=*j*} is an indicative function, and the value rule is 1 {expression with true value} = 1, 1 {expression with false value} = 0.

## 4. Experimental Data and Observations

### 4.1. General Information

86 patients with spinal fusion treated in our hospital from May 2018 to May 2020 were selected. Inclusion criteria are as follows: meet the clinical diagnostic criteria of various lumbar diseases; choose to receive spinal fusion; the fused segment is a single segment; American Society of Anesthesiologists (ASA) grade ≤ grade II; normal verbal communication skills; and informed consent to the study. Exclusion criteria are as follows: unable to tolerate surgery and anesthesia; previous history of chronic pain; test drug allergy; long-term use of opioids; with active peptic ulcer; and also participate in other studies. 86 patients were randomly divided into the control group and the multimodal group, with 43 cases in each group. There were 25 males and 18 females in the control group; the age ranged from 41 to 74 years, with an average of 58.36 ± 4.25 years; the course of disease ranged from 5 months to 9 years, with an average of 4.14 ± 1.25 years; disease types are as follows: 27 cases of lumbar disc herniation, 11 cases of spondylolisthesis, and 5 cases of lumbar spinal stenosis; fusion segments are as follows: lumbar 2–3 in 3 cases, lumbar 3–4 in 6 cases, lumbar 4–5 in 31 cases, and lumbar 5 ∼ sacral 1 in 3 cases. There were 23 males and 20 females in the multimodal group; the age ranged from 39 to 75 years, with an average of 57.19 ± 4.51 years; the course of disease ranged from 6 months to 10 years, with an average of 4.52 ± 1.38 years; disease types are as follows: 24 cases of lumbar disc herniation, 12 cases of spondylolisthesis, and 7 cases of lumbar spinal stenosis; fusion segments are as follows: there were 5 cases in lumbar 2–3, 7 cases in lumbar 3–4, 27 cases in lumbar 4–5, and 4 cases in lumbar 5 ∼ sacral 1. There was no significant difference in general data between the two groups (*P* > 0.05).

The article "Study on Automatic Multi-Classification of Spine Based on Deep Learning and Postoperative Infection Screening" was retracted in 2023. Reasons: signs of a paper mill; suspected computer-generated content; unreliable results or conclusions; lack of ethics approval or compliance.

### 4.2. Proposed Method

Both groups of patients were treated with spinal ablation by the same surgical team, and anesthesia was implemented according to the unified standard. The control group was given routine analgesic nursing, without using analgesic drugs in advance before operation, indwelling patient-controlled intravenous analgesia pump after operation, intravenous morphine analgesia within 48 hours after operation, and oral opioid analgesia when the patient complained of pain. The multimodal group was given multimodal analgesic nursing, as follows.

The patients were given preemptive analgesia before operation. The patients were given oral cimicoxib 12 hours before operation. After operation, the patient-controlled morphine analgesia pump was applied intravenously for 48 hours. Parecoxib was injected intravenously every 12 hours. After 48 hours, celecoxib was taken orally twice a day for 3–12 days. During the medication period, drug monitoring was strengthened, adverse reactions were found in time and treated accordingly, the pain law of patients is closely observed, their pain changes are evaluated, and the medication dose is reasonably adjusted, so as to achieve the best analgesic effect with the minimum dose.

### 4.3. Observation Index

1. Pain control effect: the visual analog score (VAS) was used to evaluate the pain control effect. The patients were asked to select the corresponding score according to their own pain perception. The total score was 0–10 points. With the increase in the score, the pain also increased. The patients were evaluated once at 2 h, 6 h, 12 h, 24 h, and 48 h after operation.
2. Pain control satisfaction: referring to relevant literature [4], the self-made pain control satisfaction questionnaire for spinal ablation patients was used to investigate the pain control satisfaction of patients one day before discharge. The questionnaire includes four dimensions: analgesia education, pain relief, psychological comfort, and care received, with a total of 25 items, and each item is scored 1–4 points, 4 points mean very satisfied, 3 points mean satisfied, 2 points mean generally satisfied, 1 point means dissatisfied, and the total score is 100 points. The higher the score, the higher the satisfaction with pain control. Cronbach's *α* coefficient is 0.876.

The article "Study on Automatic Multi-Classification of Spine Based on Deep Learning and Postoperative Infection Screening" was retracted in 2023. Reasons: signs of a paper mill; suspected computer-generated content; unreliable results or conclusions; lack of ethics approval or compliance.

## 5. Results

After multimodal analgesia nursing, the VASs of the multimodal group at different time points were significantly lower than those of the control group (*P* < 0.05). The difference was statistically significant, as shown in Table 1.

After multimodal analgesia nursing, the satisfaction score of pain control in the multimodal group at discharge was significantly higher than that in the control group (*P* < 0.05). The difference was statistically significant, as shown in Table 2.

## 6. Model Experiment and Result Analysis

### 6.1. Data Set

To verify and test the performance of IFS net model, the international universal data set of spinal foraminal stenosis znxtxb-14-4-hongyanfeis was selected as the test data set. The data set contains 406 intervertebral foramen images collected from spinal images of 110 clinical subjects.

### 6.2. Evaluation Criterion

 NR evaluates the multi-classification performance of machine learning algorithm in medical image data set. There are two evaluation methods based on patient level and image level. Because the IFSI data set is based on the image level, this study evaluates the recognition rate of the algorithm from the image level. Assuming the total number of images in the image verification set or test set, if the images are correctly classified, the accuracy RR at the image level is as follows:

(5) $$\begin{array}{c} \text{RR}=\frac{N_{r}}{N_{\text{all}}}. \end{array}$$

Because the accuracy is no longer the only evaluation index in the multi-classification problem, this study introduces F score as another index to evaluate the model. The two values closely related to F score are accuracy *P*_*r*_ and recall *R*_*c*_, respectively:

(6) $$\begin{array}{c} P_{r}=\frac{\text{TP}}{\left(\text{TP}+\text{FP}\right)},\\ R_{c}=\frac{\text{TP}}{\left(\text{TP}+\text{FN}\right)}, \end{array}$$

where TP is the number of true-positive records; FN is the number of false-negative records; and FP is the number of false-positive records.

As a comprehensive index of reconciliation accuracy and recall rate, F score is calculated as follows:

(7) $$\begin{array}{c} F_{\beta }=\frac{\left(\beta^{2}+1\right)}{\beta^{2}P_{r}+R_{c}}. \end{array}$$

In addition, *β* is used to adjust the ratio of the two parts. When *β* = 1, equation (8) degenerates into a simple harmonic average function, which is called F_1_ − score:

(8) $$\begin{array}{c} F_{1}=\frac{2P_{r}R_{c}}{P_{r}}+R_{c}. \end{array}$$

The article "Study on Automatic Multi-Classification of Spine Based on Deep Learning and Postoperative Infection Screening" was retracted in 2023. Reasons: signs of a paper mill; suspected computer-generated content; unreliable results or conclusions; lack of ethics approval or compliance.

### 6.3. Comparative Experiment

To verify the effectiveness of this model, this study uses the traditional machine learning algorithm to classify the IFSI data set. Traditional machine learning algorithms mainly include two steps: feature extraction and classification. In the part of feature extraction, this study selects five most advanced global algorithms for texture representation, namely local binary patterns (LBPs) [2], local phase quantization (LPQ) [12], gray-level co-occurrence matrix (GLCM) [3], histogram of oriented gradient (HOG), and oriented fast and rotated brief (ORB) [4]. The feature dimensions of the five feature descriptors are shown in Table 3.

In this study, four different classifiers are used to evaluate the above feature sets: k-NN [5], extreme learning machine (ELM) [6], support vector machine (SVM) [7], and random forest algorithm (RF) [8].

### 6.4. Experimental Result

#### 6.4.1. Performance Comparison Results of IFS Net and Traditional Machine Learning Algorithms

To verify the multi-classification performance of this algorithm on the IFSI data set, it is compared with four representative traditional machine learning classifier algorithms (k-NN, elm, SVM, and RF). The experimental results are shown in Table 4. In the two evaluation indexes of test set accuracy and F1, the result of IFS net algorithm model designed in this study is obviously better than that of traditional machine learning algorithm. From the comparison chart of classification accuracy of traditional machine learning algorithm (feature descriptor + classifier) in Figure 2, it can be seen more intuitively that in the traditional machine learning method, the selected feature vectors show stable and close results in classification performance, and the difference in recognition rate of each feature descriptor of the four traditional classifiers is within 4%. It is worth mentioning that although ORB is a key descriptor and is usually used for object recognition, it obtains better results than traditional texture features in micro-image classification.

#### 6.4.2. Performance Comparison Results between IFS Net and Other Deep Learning Algorithms

The classification performance of this algorithm and other typical deep learning algorithms on the IFSI data set is compared, and the experimental results are shown in Figure 3. In the experiment, the classification accuracy of IFS net is 87.5%, which is obviously better than other deep learning algorithms. The figure also intuitively shows that the verification set and test set of the algorithm in this study have almost the same accuracy, which shows that IFS net model has strong generalization and the ability to avoid overfitting. Due to the limitation of data set, a convolutional neural network with too deep layers does not show hierarchical advantages in the IFSI data set. For example, the serious overfitting phenomenon of GoogLeNet model is caused by its too complex structure, which is also a reason why this study adopts a relatively simple network structure. In addition, the classification accuracy of transfer learning + fine-tuning training strategy is 2.5% higher than that of self-training. As shown in Figure 4 of comparison of fitting degree of loss curves of different models, it can be seen from the train loss and val loss curves of IFS net and IFS net + TL models that the overfitting degree of the model can be reduced using the transfer learning method.

The article "Study on Automatic Multi-Classification of Spine Based on Deep Learning and Postoperative Infection Screening" was retracted in 2023. Reasons: signs of a paper mill; suspected computer-generated content; unreliable results or conclusions; lack of ethics approval or compliance.

#### 6.4.3. Analysis Results of Stenosis Recognition of IFS Image

To further test the performance of IFS net algorithm in stenosis recognition and analysis, this study conducted different IFS image stenosis recognition and analysis test experiments on the IFSI data set. The experimental results are shown in Table 5. The experimental results show that IFS net algorithm has the highest discrimination between level 0 and level 3 in the IFSI data set, and the classification result of level 1 is poor. The main reason is that the intervertebral foramen in the level 1 image is a mild mouth stenosis caused by fat occlusion in two opposite directions (vertical or transverse), which does not show the morphological changes in nerve roots [20], so it is easy to be wrongly divided into C0 (normal class). In addition, although the level 2 intervertebral foramen does not show morphological changes, the changes in its surrounding structure enable the algorithm to mine potential features and carry out correlation modeling for features to achieve accurate classification, which shows that this model has the ability to extract the features of small lesions and can establish a special relationship between the “symptom” features of different levels of diseases and IFS classification of “pathological” connection.

## 7. Discussion

Pain is a common problem after orthopedic surgery. Although sufficient postoperative analgesia has attracted enough clinical attention, 75% of patients still need to bear varying degrees of acute pain after surgery, which is extremely unfavorable to postoperative rehabilitation [4]. Therefore, how to effectively relieve the pain response after spinal fusion has become the focus and difficulty of clinical nursing. Multimodal analgesia is a new analgesic model, which mainly gives play to the superposition or synergy of analgesia through the combined use of a variety of drugs or technologies with different analgesic mechanisms, so as to reduce the dosage of a single analgesic drug and reduce the adverse analgesic reactions [5]. Studies have shown that [2] when patients undergoing spinal fusion were given multimodal analgesia during the perioperative period, the VAS at different time points after operation was significantly lower than that of the previous use of patient-controlled intravenous analgesia pump alone (*P* < 0.05). This is consistent with this study. After giving multimodal analgesic care to the multimodal group, the VASs of the multimodal group at different time points after operation were significantly lower than those of the control group (*P* < 0.05).

The article "Study on Automatic Multi-Classification of Spine Based on Deep Learning and Postoperative Infection Screening" was retracted in 2023. Reasons: signs of a paper mill; suspected computer-generated content; unreliable results or conclusions; lack of ethics approval or compliance.

It can be seen that the analgesic effect of multimode analgesic nursing is very significant. According to the usual analgesic nursing, we did not use analgesic drugs in advance before operation. After operation, we routinely indwelling analgesic pump and giving drugs on demand. Although it can alleviate the degree of pain to a certain extent, the effect has certain limitations. In the study, we gave advanced analgesia before operation to effectively avoid the transmission of noxious stimulation to the center and reduce the dosage of postoperative central analgesic drugs, After operation, a variety of drugs were used for analgesia, and the drugs were given on time to give full play to the synergistic effect of different drugs, effectively enhance the analgesic effect, and reduce the postoperative pain response. Cold therapy is a common physical therapy. Cold therapy and analgesia nursing for patients every 4 hours after spinal fusion are helpful to slow down the blood flow of local skin and slow down or eliminate the transmission of pain signals, so as to improve the pain threshold, reduce local inflammatory reaction, and reduce local pain [6].

Satisfaction is an important index to evaluate the nursing effect. Due to the single form of routine analgesia nursing, and ignoring the impact of patients' pain cognition and mental and psychological factors on the pain control effect, nursing satisfaction is not good [7].

In this study, after the multimodal analgesia nursing was given to the multimodal group, the pain control satisfaction score of the multimodal group at discharge was significantly higher than that of the control group (*P* < 0.05). In the study, we pay attention to the analgesic education of patients, clarify the relationship between mental and psychological factors and pain, fully meet the emotional needs of patients, effectively reduce or eliminate the emotional obstacles of patients, and improve the satisfaction of analgesic education and psychological comfort. In addition, music analgesia is a common nondrug analgesic method, which can play a dual role of physics and psychology in clinical application. Physically, the unique acoustic vibration of music can directly act on the corresponding nervous system in the brain, adjust autonomic nerve function, and stimulate pituitary secretion and enkephalin release, so as to inhibit adjacent pain centers. Psychologically, listening to music can arouse patients' positive and healthy emotions, stimulate human body's special emotional experience, make patients feel relaxed physically and mentally, and reduce patients' sensitivity to pain after operation [8]. In the study, according to the music preference of patients, we began to implement music analgesia on the first day after operation. Through the unique physical and psychological effects of music, we can block the mechanism of postoperative pain from physiological and psychological ways and maximize the satisfaction of pain reduction and care.

The article "Study on Automatic Multi-Classification of Spine Based on Deep Learning and Postoperative Infection Screening" was retracted in 2023. Reasons: signs of a paper mill; suspected computer-generated content; unreliable results or conclusions; lack of ethics approval or compliance.

In conclusion, multimodal analgesic care for patients undergoing spinal fusion can effectively reduce the degree of postoperative pain and improve the effect of pain control and satisfaction with pain control, which is worthy of promotion.

## 8. Conclusion and Future Work

Machine learning is a basic discipline of artificial intelligence. In recent years, due to the development of medical information engineering and the rise of big data research, medical data sets have increased explosively. A large number of medical data resources provide a research basis for intelligent machine learning. The medical industry has become one of the most transformative fields of artificial intelligence, and with broad prospects and development space, intelligent medicine not only solves the problems of insufficient resources and unequal distribution in the medical industry, but also brings a lot of entrepreneurial and business opportunities to the society. In view of the high incidence and severity of spinal diseases, this study uses the known training data set and perceptron machine learning algorithm to build an intelligent diagnostic model to realize the rapid auxiliary diagnosis of spinal diseases, greatly reduce the training cycle, and effectively improve the diagnostic accuracy. However, the research also has some defects. For example, because medical data pay great attention to patient privacy, the amount of training set data is not large enough, resulting in inaccurate model construction and so on. However, this study is intended to attract jade, which has great reference value in the intelligent development of the medical industry, can bring more intelligent applications of traditional medical diagnosis, and plays a positive role in accelerating the modernization of the medical industry and promoting the prosperity and development of medical undertakings.

The article "Study on Automatic Multi-Classification of Spine Based on Deep Learning and Postoperative Infection Screening" was retracted in 2023. Reasons: signs of a paper mill; suspected computer-generated content; unreliable results or conclusions; lack of ethics approval or compliance.

## Figures and Tables

**Figure 1:** IFS net model framework.

**Figure 2:** Comparison of classification accuracy of traditional machine learning algorithms (feature descriptor + classifier).

**Figure 3:** Comparison of algorithm performance of different depth learning models.

**Figure 4:** Comparison of loss curve fitting degree of different training strategies.

**Table 1:** Comparison of VASs between the two groups at different time points after operation ($\bar{x}\pm s$, points).

Group	N	2 h after operation	6 h after operation	12 h after operation	24 h after operation	48 h after operation
Multimodal group	43	4.34 ± 0.41	3.34 ± 0.21	3.01 ± 0.21	2.49 ± 0.21	2.11 ± 0.14
Control group	43	5.31 ± 0.37	4.98 ± 0.34	4.24 ± 0.28	3.41 ± 0.24	2.48 ± 0.23
T value		4.459	5.126	6.198	5.126	4.480
*P* value		0.035	0.026	0.013	0.024	0.034

**Table 2:** Comparison of pain control satisfaction scores between the two groups at discharge ($\bar{x}\pm s$ points).

Group	N	Analgesic education	Pain relief	Psychological comfort	Care received	Total score
Multimodal group	43	22.36 ± 1.26	22.56 ± 1.23	22.39 ± 1.87	22.41 ± 1.42	90.41 ± 6.25
Control group	43	17.26 ± 1.11	17.39 ± 1.29	17.26 ± 1.99	17.29 ± 1.36	70.26 ± 3.29
T value		6.654	7.111	8.274	6.051	7.862
*P* value		0.010	0.008	0.004	0.014	0.005

**Table 3:** List of feature descriptors and their feature vector dimensions.

Descriptor	Eigenvector dimension
LBP	59
LPQ	256
GLCM	8
HOG	4356
ORB	32

**Table 4:** Accuracy and *F*_1_ statistics of different methods.

Traditional classifier	Method	Validation set accuracy	Test set accuracy	*F*_1_
1-NN	LBP	49.4 ± 2.1	51.8 ± 2.5	0.712
	LPQ	63.5 ± 2.7	53.7 ± 2.7	0.517
	GLCM	65.3 ± 1.7	53.6 ± 1.6	0.725
	ORB	66.1 ± 3.5	63.7 ± 3.4	0.764
	HOG	51.7 ± 1.3	61.3 ± 0.7	0.768

ELM	LBP	69.4 ± 1.0	51.3 ± 2.1	0.742
	LPQ	61.6 ± 1.8	57.6 ± 2.3	0.76
	GLCM	73.3 ± 2.9	57.3 ± 3.0	0.786
	ORB	67.2 ± 1.9	65.4 ± 3.8	0.73
	HOG	63.5 ± 2.7	61.4 ± 1.8	0.697

**Table 5:** Confusion matrix of stenosis classification results of IFS net algorithm.

Stenosis category	*C*_0_	*C*_1_	*C*_2_	*C*_3_	ACC/%
*C*_0_	24	0	0	2	92.31
*C*_1_	4	16	3	3	71.54
*C*_2_	4	0	21	0	84
*C*_3_	0	0	3	22	88

## Data Availability

The data sets used during this study are available from the corresponding author on reasonable request.
